# Occupational Therapy-Based Energy Management Education in People with Post-COVID-19 Condition-Related Fatigue: Results from a Focus Group Discussion

**DOI:** 10.1155/2022/4590154

**Published:** 2022-04-14

**Authors:** Ruth Hersche, Andrea Weise

**Affiliations:** Rehabilitation Research Laboratory 2rLab, Department of Business Economics, Health and Social Care, University of Applied Sciences and Arts of Southern Switzerland, Manno/Landquart, Switzerland

## Abstract

Persons with post-COVID-19 conditions have prolonged symptoms and longer-term consequences which can prevent them from returning to previous everyday functioning. Fatigue is the most frequent symptom reported in literature. Occupational therapists (OTs) are specialized in client-centered problem analysis, counseling, and education to recover occupational engagement and performance in everyday life. Since the beginning of the COVID-19 pandemic, OTs have been challenged to respond with services adequate to the needs of this patient group. Energy management education (EME) was initially developed for persons with multiple sclerosis-related fatigue and then made independent of diagnosis suitable to persons living with chronic disease-related fatigue. EME, a structured self-management education, is becoming a part of the new services. This study was aimed at exploring the initial experiences of OTs using the EME protocol and materials with persons with postacute COVID-19 and/or post-COVID-19 condition-related fatigue and gathering their recommendations for improvements and adaptions. One online focus group discussion took place in May 2021 with OTs experienced in using the EME protocol. The topics addressed were the institutional context of the OTs and their experiences during the treatment. A thematic analysis was performed. According to nine OTs working in different settings in Switzerland, the EME protocol is exploitable in both in- and outpatient settings and was judged appropriate by them, even if the EME materials can be improved. The main challenges for the OTs were the short period their patients had lived with fatigue; the discrepancy between self-concept, self-perception, and performance; and the insecurity, fear, and anxiety related to recovery. Further research is needed to include the perspective of EME participants and to measure quantitative outcomes such as fatigue impact, self-efficacy, occupational performance, and quality of life. Until the existing EME protocol is improved, it is applicable to persons with post-COVID-19 condition-related fatigue.

## 1. Introduction

Severe acute respiratory syndrome coronavirus 2 (SARS-CoV-2) is the pathogen responsible for the coronavirus disease 2019 (COVID-19) pandemic, which has resulted in a global health care crisis and strained health resources worldwide [1]. COVID-19 is now recognized as a multiorgan disease with a broad spectrum of manifestations [2]. While the population of patients recovering from COVID-19 is growing, evidence indicates the infection can have prolonged effects and longer-term consequences [3], which prevent returning to pervious life routines, performance, and work [4]. Signs and symptoms that develop during or after an infection consistent with COVID-19, beyond 4 weeks from the onset of symptoms, are currently defined as postacute COVID-19, and those ongoing after 12 weeks, not explained by an alternative diagnosis, are defined by WHO consensus as post-COVID-19 condition and known as long COVID [5]. A prevalence study in UK showed that fatigue was the most common symptom (43%) reported as part of an individuals' experience of long COVID, followed by shortness of breath (32%), muscle ache (25%), and difficulty concentrating (23%) [6]. Fatigue emerges independent of the severity of initial infection and is a common COVID-19 sequelae in adults aged less than 50 years [4]. Data from the Zürich SARS-CoV-2 population-based cohort study (*n* = 431) [3] reports that 26% of individuals had not fully recovered within 6 to 8 months of SARS-CoV-2 infection, with 55% of study participants experiencing fatigue, 25% experiencing dyspnea, and 26% experiencing depression.

Fatigue is a complex, multicausal, multidimensional, and nonspecific phenomenon with high prevalence after acute viral infection, neurological diseases, and chronic long-term conditions [7]. The term “fatigue” describes the difficulty or inability to initiate activity (subjective sense of weakness); reduced capacity to maintain activity (easy fatigability); or difficulty with concentration, memory, and emotional stability (mental fatigue) [7]. Fatigue is a significant burden influencing occupational performance, family work, and lifestyle. This results in specific health care needs of the working population with post-COVID-19 condition-related fatigue to which the health care system needs to respond.

The Swiss health care system is currently developing therapeutic services for this group of patients [8]. The primary goal of occupational therapy (OT) in persons with fatigue is to enable participation in daily activities through behavior changes and to support occupational performance in all significant life areas and to enable self-determination, well-being, and health. Fatigue self-management education delivered in peer-groups or individual sessions has shown positive effects on the impact of fatigue, occupational performance, and quality of life (QoL) in persons with multiple sclerosis [9], cancer survivors [10], infectious diseases like systemic lupus erythematosus [11], or rheumatoid arthritis [12]. Despite this evidence, structured and systematic fatigue self-management education was not part of OT practice in Switzerland and neighboring countries until 2017 owing to a lack of culturally appropriate and feasible treatment materials. The first step to bridge this gap was to develop an inpatient energy managing education for persons with MS-related fatigue [13]. This treatment protocol is rooted in evidence-based intervention protocols for energy conservation [14] and cognitive behavior therapy approaches [15, 16]. In 2018, a small-scale RCT has confirmed pertinence and feasibility of the inpatient energy management education (EME) and has shown small to medium effects on occupational performance, self-efficacy, and quality of life [17].

The strategies taught during EME are disease unspecific; therefore, the inpatient EME manual and workbook was subsequently adapted into a disease-independent version. This version is based on best practice recommendations and scientific evaluations of disease-specific protocols for different populations, such as cancer [17, 18], rheumatoid arthritis [12], stroke [19], heart failure [20], chronic pulmonary obstructive disease [21], spinal cord injury [22], traumatic brain injury [23], systemic lupus erythematosus [11], and Parkinson disease [24]. It has been evaluated during a pilot study in 2018, by a group of Swiss OT experts from different fields [25]. This enabled the creation of mixed patient groups, especially relevant in the outpatient setting, and has facilitated broad access to group OT interventions for people living with fatigue owing to a chronic condition or after a disease.

The goal of EME is to ensure that participants learn to manage their available energy to achieve a satisfying and meaningful daily routine. Participants acquire understanding about factors that influence their level of energy and the skills to conserve and manage it by using behavioral strategies. Subsequently, they identify and implement tailored behavior modifications and adapt their habits and routines. The EME manual for OTs provides detailed information for each lesson and supports the OT during face-to-face interactions. The EME workbook for participants summarizes the information from each lesson in a costumer-adapted way and provides the worksheets and the self-training tasks used during and between the lessons. The outpatient and inpatient versions of EME are based on the same literature, consists of the same eight topics, and use the same behavior change techniques. They differ in frequency of lessons and self-training tasks owing to the different settings in which they are delivered (Table 1). The inclusion criteria are as follows: experienced in living with fatigue (FSS, score ≥ 4; [26]), no major depression (BDI-FS, <8; [27]), no major cognitive impairments (MOCA, ≥26; [28]), sufficient linguistic ability, and motivation for self-management education, which are assessed during an interview by the OT before starting EME.

Since 2019, about 130 OTs from Switzerland, Austria, Germany, Italy, and Luxembourg have participated in a 2-day introduction course in leading EME groups. A first update and network meeting of trained EME OTs took place in the summer of 2020 via online conference. Since January 2021, an increasing number of OT departments has been asked to treat people with postacute COVID-19 and/or post-COVID-19 conditions in different settings (acute inpatient, inpatient rehabilitation, and outpatient reintegration). They are challenged to define treatment contents, delivery modalities, and services in coordination with other disciplines for the needs of this new patient group. Some of the EME-trained OTs have started to include persons with post-COVID-19 condition-related fatigue into their mixed EME groups or have used the EME materials as part of individual therapy. It is important to collect their clinical experiences and to share it with other OTs that are searching for feasible and appropriate treatment programs to implement in their care settings.

This focus group study was aimed at exploring the experiences of OTs using the EME treatment protocol and materials with persons with postacute COVID-19 and/or post-COVID-19 condition-related fatigue and collecting their recommendations for improvements and adaptions.

### 1.1. Materials and Methods

Focus group research is “a way of collecting qualitative data, which—essentially—involves engaging a small number of people in an informal group discussion (or discussions), ‘focused' around a particular topic or set of issues” [27]. An expert moderator that stimulates in an open atmosphere, perceptions, ideas, opinions, and thoughts leads the discussion [28]. We followed a widely accepted systematic process for data collection, data handling, and data analysis based on McLennan et al. [28]. The focus group was led by the developers of EME (RH and AW). They are experienced OTs, used to leading groups, and skilled in qualitative research methods, as focus group interviews, to explore the experiences of deliverers and consumers of health care services.

A convenience sample of Swiss OTs (*n* = 105) who had attended an EME course since 2018 was notified via e-mail (EME mailing list) about the online 1.5-hour focus group and asked to contact AW or RH if interested in attending. The following inclusion criteria were adopted: (1) completed an EME course or experience with EME in daily practice, (2) experience in treating people with postacute COVID-19 or post-COVID-19 condition-related fatigue or prepared to do so in the near future, and (3) consented to audio recording of the focus group discussion.

The interview guide was developed in partnership by AW and RH and consisted of an entry, a main, and a conclusion phase and two subjects: (1) institutional contexts in which EME is a planned or an already implemented service for people with postacute COVID-19 and/or post-COVID-19 condition and (2) experiences in using EME in people with postacute COVID-19 and/or post-COVID-19 condition-related fatigue or rather in using it for preparing services for this patient group. The focus group started with a presentation of the aim and the purpose of the focus group, the involved participants, and their clinical settings. In the main section, five open-ended questions were discussed. The first four questions were oriented on the treatment process (assessment procedures, main restrictions experienced by patients, treatment, and outcomes) while the last question regarded suggestions and recommendations from OTs regarding EME in people with postacute COVID or post-COVID-19 condition. AW conducted the entry and conclusion phase, and RH led the central part of the discussion. To encourage sharing experiences and the identification of emerging subjects, the researchers used specification questions. Throughout the whole discussion, the comoderator took field notes of nonverbal communication elements and key statements. At the end of the focus group, AW summarized to verify the key elements of the discussion and to animate the participants to reflect on the completeness of the collected data or rather to add missing elements. Immediately after, RH and AW made a debriefing. The online discussion and the debriefing were audiorecorded and transcribed word-for-word by RH and compared by AW with her field notes and completed where necessary.

Subsequently, a thematic analysis in six steps was performed by RH [29]. After getting familiar with the data, initial codes were generated. Subsequently, the codes were collapsed under labels and categories. The themes were searched with a deductive approach. Additional themes that arose were inductively built and integrated. Then, the themes were reviewed and defined by RH and AW. A report containing findings and recommendations was sent to the focus group participants for member checking.

## 2. Results

### 2.1. Participants

Nine OTs working in different clinical settings and parts of Switzerland have participated in the online focus group in May 2021, which had a duration of 1.50 h and was performed in German language. All participants were experienced in using EME with persons with different chronic conditions (see Table 2).

### 2.2. Themes

There were five consistent themes identified: (1) changed and additional demand for occupational therapy-based energy management education, (2) referral and access to EME of persons with post-COVID-19 condition-related fatigue, (3) differences compared to other groups of patients living with fatigue, (4) experiences and outcomes of using EME materials, and (5) recommendations to the EME developers. Theme 1 shows the response of institutions to the new treatment needs at the macrolevel of the health system. The implementation and the access organization (2) and the recommendations for the EME developers (5) regarded both the mesolevel. Themes 3 and 4 belong to the microlevel because they were related directly to the clinical experiences and were discussed only by the six participants with experiences with EME with this new patient group.

#### 2.2.1. Changed and Additional Demand for Occupational Therapy-Based Energy Management Education

The institutions in which the focus group participants are active are different in their mandate, dimension, catchment area, and client groups. At one public hospital, EME was used primarily with people with chronic pain in a one-to-one setting (outpatients). Their neurology department had recently started to refer also persons with post-COVID-19 condition-related fatigue to their OT service. In another hospital, OTs had established mixed outpatient EME groups with patients, which were referred by internal physicians (fatigue consultations at the psychiatric outpatient department, mainly chronic fatigue syndrome). More recently, persons with post-COVID-19 condition-related fatigue have been integrated into these EME groups. Due to the high demand, they offer now additional EME groups only to persons with post-COVID-19 condition-related fatigue.

*Originally, we conducted the EME for persons with rheumatoid diseases. Now, also Long Covid patients joined, in mixed groups. Meanwhile there are also groups with only patients with Long Covid.* (OT9)

Three OTs were employed in private rehabilitation clinics. One OT treated primarily persons with postacute COVID-19 neurological sequelae. In the other two clinics, inpatient EME groups with mixed diagnostic patients including persons with postacute COVID-19 and post-COVID-19 condition-related fatigue were part of the rehabilitation program. One OT treated postacute COVID-19 patients with fatigue in an individual setting and integrated EME content and materials into the occupational therapy treatment. One focus group participant was an independent OT with her occupational therapy practice. She worked mainly in a home setting with people with cognitive impairments due mainly to neurological diseases, where the effects of fatigue were addressed with a patient-tailored choice from the EME materials. She reported that the referrals for OT from inpatient rehabilitation clinics (neurology departments) seem to increase due to persons with post-COVID-19 condition. One OT was employed by an organization that owns several outpatient OT centers in the German part of Switzerland. Mixed outpatient EME groups for persons with chronic conditions were prepared to be implemented in spring 2021. All participants agreed that the demand for OT for persons with post-COVID-19 condition is slowly increasing, and that they are expecting this trend to continue.

#### 2.2.2. Referral and Access to EME of Persons with Post-COVID-19 Condition-Related Fatigue

All except two OTs receive a general referral for OT treatment without specific program indications for patients with postacute COVID-19 or post-COVID-19 condition with occupational performance problems. It is, according to the regulations in Switzerland (freedom of and responsibility for methods used in the OT treatment), up to them to suggest EME after assessment of the occupational performance needs and priorities of the patients.

*Indirect access to EME*. In this standard case, the OTs reported that the assessment procedure did not differ from other patients they had worked with. During the initial interview, they assessed current occupational problems, the occupational and medical history, occupational performance (e.g., COPM [30] and OSA [31]), and context factors. The majority of OTs addressed the issue of fatigue only when they knew the person a little better, when they suspected a high impact of fatigue on daily life, and that the issue of energy management might be important. In such cases, they use questionnaires to assess fatigue (e.g., fatigue impact scale [32] or fatigue severity scale [26]). They highlighted the importance to consider (by subjective valuation or screening instrument) the cognitive abilities and the motivation before proposing an EME group as a treatment option.

*Direct access to EME*. In this special case, patients were screened by the physicians for EME inclusion criteria and informed about EME before being referred to the OT. Then, OTs contacted the person by phone to explain the aims and contents of EME once again. The OTs affirmed that this preamble is necessary to make sure that the patients are qualified for the group.

*Because physicians explain sometimes rudimentary, some people say they had imagined something else, e.g. respiratory therapy and endurance sports, so it becomes clear that they are not qualified for the group*. (OT3)

If interested and includable, patients can start within the next available EME group, in which OSA and SEPECSA [33] are integral assessments of the first lesson.

Independently from the institution and the type of access, the OTs agreed that it is crucial to explain the aims of EME and to clarify the expectations of the patients before starting with the program.

#### 2.2.3. Differences Compared to Other Groups of Patients Living with Fatigue

The six OTs with experience in treating persons with postacute or post-COVID-19 agreed on the observed functional restrictions and limitations in everyday life. They reported that there are differences compared to persons living with other chronic disease-related fatigue they had worked with previously.

The OTs agreed that the spectrum of limitations experienced by persons with post-COVID-19 was very broad and individual, including and combining decreased physical and cognitive functions. OTs working in the inpatient setting reported more limitations on body function (e.g., shortness of breath, decreased oxygen saturation and attention, and increased anxiety and insecurity) and activity level, while those working in the outpatient setting also reported limitations in different occupational areas.

*There are the patients who cannot concentrate cognitively at all, and are extremely sensitive to light and noise, but also the opposite, people who are very limited physically but have no problems mentally, and everything in between.* (OT5)

*Lack of attention, but also being able to stay awake, being physically present, and not falling asleep in the chair are big issues*. (OT2)

Several OTs reported that EME participants with post-COVID-19 condition often experience themselves as extremely impaired in the area of work, family activities with young children, school, or studies. Patients more frequently declared the loss of leisure and social activities, while self-care was a less prominent therapeutic subject.

*2.5-hour long working sessions with the boss, those are such issues* (OT2)

*Young adults who are active, who have lots of different hobbies and are always booked up and suddenly find a weekend with friends to be mega exhausting* (OT3)

The focus group participants agreed that persons with postacute or post-COVID-19 condition have great difficulties in recognizing their own physical and cognitive limits. They described that their patients experienced a great uncertainty on their performance limits and difficulties of self-perception and that they often are experiencing a depressed mood. The OTs agreed that patients are far from accepting post-COVID-19 condition consequences, which is different from people with chronic diseases who are more advanced in the process of acceptance and adaptation.

*Being pulled out of an 80% job and now only being able to work a few hours a week is hard bread for many* (OT9)

*They are more susceptible to not recognizing their own limits, there is a greater risk that they will overstep these limits and will continue to do so (…), while other groups of patients have realized their limits for a long time*. (OT1)

One OT thinks that in other patient groups with chronic diseases, fatigue has an insidious effect on everyday life. In comparison, persons with post-COVID-19 condition-related fatigue experienced sudden and incisive limitations in everyday life.

*Fatigue is suddenly there or suddenly still there*. (OT1)

The average age of EME participants with post-COVID-19 condition seemed to be lower compared to EME participants with other diseases they had included in EME groups previously.

#### 2.2.4. Experiences and Outcomes of Using EME Materials

The six OTs with experience in treating persons with postacute or post-COVID-19 agreed on a general appropriateness and relevance of the whole content of the EME program for this group of patients.

*We actually implement it one-to-one, the whole program!* (OT3)

W*e do not follow the program and we do not do it in a group, but we use all parts of it*. (OT2)

In the discussion, the lessons “energy account,” “break management,” “occupational balance,” and “effective communication” took more space while the topic “body and environment” and “simplifying activities” were less often mentioned. From the OTs' perspective, the first lesson that provides information about fatigue seemed to be especially important because persons with postacute COVID-19 or post-COVID-19 condition-related fatigue often had very little knowledge compared to patients with chronic diseases.

*To realize during the first lesson, that fatigue can also be cognitive is for many very educational* (OT4)

The lesson “break management,” which includes daily scheduling, and the lesson on “occupational balance,” which includes weekly scheduling and with a priority list, were highlighted for their relevance by the OTs. They agreed that these instruments helped to make plan for the time after discharge and slowly increase the activity level in daily life. Energy profiles were also mentioned as a strategy to promote self-awareness and served as feedback. This tool can be easily integrated in the therapeutic processes also with individual sessions when patients cannot follow the whole EME program.

*The energy account, I always bring that. It's very insightful, super example, patients find it very understandable* (OT1)

OTs defined the lesson “effective communication” as a key issue. In this lesson, they train communication skills around fatigue that are especially important in the areas of work and social activities.

*Outcome evaluation*. To evaluate the outcomes of EME, OTs refer to their observations and feedback from participants in addition to the scores of the assessment results. The OTs affirmed that they observed sometimes positive changes in EME participants (e.g., knowledge on fatigue, consciousness on energy level, and confidence on personal skills in managing their daily routines) or they receive individual feedbacks and reactions, which varied from “it was ok” to “very positive.” Some participants were relieved and grateful that the EME group existed. In other, but rather rare cases, patients were rather unsatisfied.

*Someone say that EME is his weekly highlight* (OT2)

*Until now, I remember only one person who was very unsatisfied* (OT9)

Standardized feedback to the referring physician is not yet the norm. Often EME participants have scheduled appointments with their physician and use these meetings to give verbal feedbacks about their outcomes. In one institution, the OT integrated the outcomes in the final report to the referring physician.

The dropout rate tended to be low. One OT hypothesized that participants who had not yet processed what had happened to them or were not emotionally stable enough to talk about fatigue, were more likely to drop out of the EME group. Other reasons mentioned were irregular working schedules of the participants or cognitive difficulties. While persons with a long experience of living with fatigue (e.g., people with MS) sometimes quit the education because they seem to know already everything about energy management, persons with post-COVID-19 condition-related fatigue did not quit the program due to that reason. OTs who offered EME in a one-to-one setting usually had no dropouts. They think it is because they can better adapt to the specific needs and issues of the individual.

### 2.3. Recommendations to the EME Developers

The focus group participants suggested structural adaptations and knowledge elements for OTs (manual) and the patients (workbook) to improve the compatibility with the needs of persons with post-COVID-19 condition-related fatigue and usability for the leading OTs (Table 3).

## 3. Discussion

This qualitative focus group study with 9 OTs experienced in energy management education and involved in preparing services for and treating persons with postacute or post-COVID-19 condition has reported relevant findings. Referral and access to EME differ between institutions. The implementation of new services is ongoing due to an increasing demand. The OTs reported limited self-perception, insecurity, and ongoing adjustment of the self-concept as important differences to persons with long-term experience with fatigue due to other health conditions. Delivery format and adherence to the EME protocol are adapted to the internal provisions, but the EME protocol and associated materials were successfully used in both inpatient and outpatient settings. Worksheets and tools were rated as applicable and adequate in clinical practice and all eight main topics as relevant and appropriate contents for this new patient population, too, but EME materials can be improved. Relevant recommendations have been made. Additionally, tasks during the lesson should support more often the reflection of the self-concept of the participants for this new patient group.

The different access modalities and delivery modalities that were described by the focus group participants showed that the Swiss health care system at that date had not yet responded nationally coordinated to the needs of persons with post-COVID-19 condition. To evolve towards a high-quality service for persons with post-COVID-19 condition, the following principles have to be reinforced; easy access, continuum of care, multidisciplinary rehabilitation, evidence-based standards, and further development of the knowledge base and clinical service like proposed in another recent study [34].

Considering the different perspectives of people with post-COVID-19 condition compared to persons with long-term experience with fatigue (e.g., chronic fatigue syndrome and multiple sclerosis) and due to the results of the focus group discussion, people with post-COVID-19 condition-related fatigue should be supported at first, during an individual contact with short and clear person-relevant information and tips (e.g., break management), like also proposed by several recent guidelines [35]. These people should only be included in EME groups if the fatigue is persisting and an advantage from a more thorough and time-consuming self-management program is expected.

The main symptoms reported by the OTs were, in addition to fatigue, limitations in cognitive functions, insecurity, acceptance, anxiety, and reduced self-perception. Essential restrictions were in work, school, and social participation. That is in line with prevalence studies of post-COVID-19 condition [34] and qualitative research [36] that highlight degrees of psychological distress and symptoms of chronic anxiety and cognitive functioning particularly related to economic hardships. During the COVID-19 pandemic, people have been exposed to an overload of information and continually searched for adequate, reliable, and recent information on their symptoms, which might have increased stress and anxiety, according to findings of a recent systematic review [37]. OTs discussed symptoms like shortness of breath or muscle ache less, probably not because not present, rather because less unexpected by the OTs.

EME is a complex group intervention with a standardized structure and a certain degree of flexibility and tailoring, which requires a high level of competence from the leading OT. This study showed that the EME material was used differently in group settings than individual therapies. Those who offered groups adhered quite clearly to the manual. Those who worked in individual settings chose client-centered content and worksheets according to the main topics of their patients. This difference can depend on different factors. First, when applying the protocol, OTs might be confronted with essential barriers on the mesolevel. Therefore, they are constrained to use the individual setting and adapt their interventions. Second, the significance of treatment fidelity might not be well recognized. Most psychosocial interventions outside occupational therapy currently rely on manualization as the critical mechanism for ensuring treatment fidelity and guaranteeing success [38]. However, only a sparse number of manualized occupational therapy interventions exist [39]. One reason for this paucity is the continuing challenge for occupational therapy researchers and developers to reconcile the client-centered and individualized nature of OT practice with the need to manualize interventions [38].

The OT-based EME is a self-management educational intervention that aims to increase resilience to cope with everyday life tasks and reestablish occupational engagement in routines and roles. An elementary aspect of achieving this goal is a positive self-concept based on self-esteem and a sense of competence [40]. Post-COVID-19 individuals experience suddenly incisive performance restrictions in everyday life owing to fatigue and other symptoms. They are confronted with discrepancies between their self-concept and responsibilities and actual self-perceptions. Together with the uncertain prognosis, this divergence may increase their fear and anxiety and depress their mood [41, 42]. Multidisciplinary rehabilitation with gradual, flexible, and cautious increases in physical and mental activity that are based on a person's energy envelope and within their limitations (e.g., activity pacing and exercise training) [43] supports the reacquisition of the perceived self-efficacy, which is the base for the implementation of behavior changes and performance recovery.

### 3.1. Limitations and Strengths

Due to scheduling and pandemic constraints and workloads of OTs, only one online focus group using convenience sampling was conducted, and therefore, saturating the data was not achieved. The interview guideline had not been piloted before. Only six out of nine OTs had practical experience in treating persons with post-COVID-19 condition, while three had prepared for it soon. Therefore, for three of the five themes of the results, the experiences of only six OTs were available. However, all were trained and experienced in energy self-management education (EME). The focus group was led by the developers of the EME, who are well-known in the Swiss-OT community. That could have created a selection and information bias. OTs with negative experiences with EME could have declined a priori to participate in the focus group; others might have been in awe to share ambiguous experiences. The two authors have performed the analysis, who could have been inclined to underline positive statements.

The next important step will be to collect and integrate the considerations and opinions of people with post-COVID-19 conditions who participated in an EME group.

## 4. Conclusion

This focus group study was aimed at exploring OTs' experiences using the EME treatment protocol and materials with persons with postacute COVID-19 and/or post-COVID-19 condition-related fatigue or of using them for preparing services for this group and for collecting their recommendations for improvements and adaptions.

The results of this first focus group discussion with nine Swiss OTs trained in EME showed that the EME protocol and its materials are adequate and applicable in an in- and outpatient setting, both in peer-groups containing only persons with postacute COVID-19-related fatigue and in groups with persons with mixed diseases that cause fatigue and in the one-on-one treatment. Therefore, EME is usable for preparing further services for this new patient group, but EME materials and training of OTs can be improved to the specific needs of this group.

During EME training for OTs, the level of treatment fidelity to the program versus flexibility and tailoring it to the specific individual's needs should be worked out more precisely and more binding. Due to the fact that persons with longer experiences with fatigue (e.g., persons with chronic diseases) are often further advanced in their experiences with the symptom and their reflections and coping strategies than this new patient group, an initial one-on-one-treatment session is highly recommended, where expectations, aims, and readiness for self-management education in a group setting should be explored. Alternatively, the individual treatment setting is an option for persons with postacute COVID-19-related fatigue that are not (yet) ready for an EME group but could benefit from elements of EME.

The introductory section of the workbook for EME participants needs to contain facts on post-COVID-19-related fatigue and related aspects. During the first lesson and repeatedly over the whole EME program, the OT can pick up open questions about the diagnosis, clarify doubts, qualify beliefs, and underline facts to support informed decision-making and communication of EME participants with post-COVID-19-related fatigue, taking into account that there is a lot of nonfiltered information and beliefs about this topic in the general population. Additional tasks about self-perception and exploring and accepting new limits (physically and cognitively) and as support for the elaboration of a new self-concept should be created, taking into account that this specific patient group is out of the sudden confronted with this and other symptoms and the consequences of it on their everyday life and roles.

Further research is needed to obtain the perspective of EME participants and revise the materials with the support of the users. After adjusting the materials, in a subsequent step, quantitative data on self-efficacy, fatigue impact, occupational performance, and quality of life after EME in persons with post-COVID-19-related fatigue should be evaluated.

## Figures and Tables

**Table 1:** Description of energy management education (EME).

Topic of lessons 1-8	Outpatient version	Inpatient version	Applied behavior change techniques
Energy account; break management; occupational balance; use of body & environment; simplifying activities; effective communication; my goals; review and reinforce	L1–7, peer-group (2–5 participants) once a week; L8 peer-group, 8 weeks after L7; duration: 75 min per lesson	L1 individual 1–3 days from admission (60 min); L2–6 in peer-group (2–7 participants) twice per week (60 min); L7 individual (30 min); reinforcement mail 8 weeks after discharge	Shaping knowledge; experience exchange & social support; feedback & monitoring; compared behavior & outcomes; goals & action planning; antecedents; self-belief

Abbreviations: L: lesson; min: minute.

**Table 2:** Characteristics of the focus group participants.

Gender: *n* (female/male)	9/0

Age: years (median/Min–Max)	44/23-58

OT working experiences: years (median/Min–Max)	12/2-26

Regions from Switzerland: *n*	
Zürich	4
Mittelland	3
Ostschweiz	1
Ticino	1

Delivery setting: *n* (inpatient/outpatient-home)	5/4

Participants experience in using EME with different patient groups: *n*	
Cancer survivors	1
Neurological diseases (e.g., MS and stroke)	5
Chronic fatigue syndrome	2
Chronic pain	1

EME with persons with postacute or post-COVID-19 condition-related fatigue: *n* (applied/not applied, but prepared to use)	6/3

**Table 3:** List of recommendations and suggestions.

*Structural adaptations*	(i) Ninety-minute duration instead of 60–75 minutes: inclusion of a break
*Knowledge elements*	(i) Update the manual and the workbook with basic facts and definitions on post-COVID-19 condition-related fatigue as well as clarify information on terms like *crash*, *postexertional malaise*, or *brain fog* to understand these phenomes better (iii) Add to the manual a paragraph on the topic of healing; from the perspective of persons with post-COVID-19 condition, this differs from that of people with chronic diseases (iv) Add instructions (manual) for OTs on how to deal with patients who still have little experience with their fatigue (v) Add short information (manual) on how insurance companies deal with reintegration or retirement with this new patient group. That will support the OTs to reduce patients' feelings of uncertainty

*New tasks*	(i) Add in lesson 6 “effective communication” a task aimed to reflect on the modified self-perception/image and its legitimization and dealing with uncertain prognosis, in relation to relatives or colleagues

*Usability*	(i) Text template for initial information for EME candidates (manual) (ii) Add in the introduction of the EME manual a clear demarcation towards other education programs, e.g., sleep-hygiene education (iii) Text template for a final report (manual)

## Data Availability

The data used to support the findings of this study are included within the article. However, for more information, requests for access to these data should be made to Ruth Hersche (ruth.hersche@supsi.ch).
